This article has been retracted.

# Expression and Possible Significance of ACE2 in the Human Liver, Esophagus, Stomach, and Colon

**DOI:** 10.1155/2021/6949902

**Published:** 2021-08-25

**Authors:** Yiwen Liu, Qing Wu, Dongmei Wan, Huiqin He, Hailian Lin, Kelang Wang, Genxiang Que, Yuanyuan Wang, Yongjun Chen, Xiaoqing Tang, Lingbo Wu, Xuefeng Yang

**Affiliations:** ^1^The Affifiliated Nanhua Hospital, Department of Gastroenterology, Hengyang Medical School, University of South China, Hengyang 421001, Hunan, China; ^2^The Affifiliated Nanhua Hospital, Department of General Practice, Hengyang Medical School, University of South China, Hengyang 421001, Hunan, China; ^3^The Affifiliated Nanhua Hospital, Department of Orthopaedic Traumatology, Hengyang Medical School, University of South China, Hengyang 421001, Hunan, China; ^4^The Affiliated Nanhua Hospital, Department of Neurology, Hengyang Medical School, University of South China, Hengyang 421001, Hunan, China; ^5^The First Affiliated Hospital, Institute of Clinical Medicine, Hengyang Medical School, University of South China, Hengyang 421001, Hunan, China; ^6^The Affifiliated Nanhua Hospital, Department of Respiratory Medicine, Hengyang Medical School, University of South China, Hengyang 421001, Hunan, China

## Abstract

Angiotensin-converting enzyme 2 (ACE2) has been identified as the key receptor of SARS coronavirus that plays a key role in the pathogenesis of SARS. It is known that ACE2 mRNA can be expressed in most organs. However, the protein expression of ACE2 is not clear yet. To explore the role of ACE2 as a precipitating factor in digestive organ damage in COVID-19, this study investigated the expression of ACE2 protein in the human liver, esophagus, stomach, and colon. The result showed that ACE2 can be expressed in the liver, esophagus, stomach, and colon, which suggests SARS-CoV-2 may enter the digestive system through ACE2 and cause liver damage and gastrointestinal damage. It is hoped that the result of the study will provide a new strategy for the prevention and treatment of digestive organ damage under COVID-19.

## 1. Introduction

Angiotensin-converting enzyme 2 (ACE2) is a kind of transmembrane protein. Its gene is situated in the X chromosome. The protein which is coded by the gene is composed of 805 amino acids, including the N-terminal signal peptide sequence in the pericellular membrane, the C-terminal sequence in the transmembrane domain, and the intracellular [1–3].

ACE2 generally plays a key role in the human body through three ways. First, it participates in the regulation process of the renin angiotensin system (RAS). The renin secreted by the periglomerular cell of the kidney can convert angiotensinogen in the blood into inactive angiotensin I (Ang I). In the plasma and tissues, especially on the surface of the vascular endothelium of the pulmonary circulation, there is ACE2 that can hydrolyze Ang I to 8-peptide angiotensin II (Ang II). Ang II plays a role in the regulation of blood pressure, proinflammatory, and apoptosis promoting through binding to the related receptors. Second, studies have revealed that ACE2 acts on the Kinin–Kallikrein system (KKS) by degrading dearginine bradykinin, a bradykinin analogue. Dearginine bradykinin can bind to the B1 receptors which are expressed in tissues. Therefore, the release of inflammatory factors is promoted, which plays an important role in the process of inflammation as increasing the production of local nitric oxide causes hemangiectasis [4, 5]. Third, ACE2 is closely associated with the incidence of severe acute respiratory syndrome (SARS) in 2003 [6, 7]. In 2003, the SARS epidemic which is caused by severe acute respiratory syndrome coronavirus (SARS-CoV) spread all over the world. Based on the fact that Vero E6 cells could be infected and replicated by SARS-CoV [8], Li's team determined that ACE2 could effectively bind the S1 domain of SARS-CoV S protein by applying the coimmunoprecipitation. Therefore, it was proved that ACE2 is the needful receptor for SARS-CoV infection because it promotes the entry of the virus through the membrane fusion mechanisms [9]. The novel coronavirus pneumonia 2019 (COVID-19) broke out in late 2019. Its pathogen is named as severe acute respiratory syndrome coronavirus (SARS-CoV-2) by the International Committee on Virology. It has triggered a global epidemic. Studies have found that SARS-CoV-2 and SARS-CoV share a high degree of similarity. Based on the fact that both of them belong to the genus *β*-coronavirus, there is 80% homology in terms of genome sequence [10]. But the ability of SARS-CoV-2 to bind the S protein and ACE2 is much stronger than that of SARS-CoV [11]. We hypothesized COVID-19 that is caused by SARS-CoV-2 had similar pathogenesis with SARS which is caused by SARS-CoV.

In the early stage of our study, we found that except the obvious damage on the respiratory organ, damage on other organs also showed in the 48 COVID-19 patients in the Hengyang area, including the digestive organs. Among the 48 patients with COVID-19, 27.1% of the patients had poor appetite, 8.3% of the patients had nausea and vomiting, and 14.7% of the patients had diarrhea. With the primary diseases of the liver, such as viral hepatitis, excluded, ALT was increased in 22.9% of patients, AST was increased in 20.8% of patients, ALP was increased in 5.4% of patients, and *γ*-GT increased in 21.6% of patients [12]. The data are accordant to the published study [13]. The clinical symptom analysis of Xie's team shows that ALT was increased in 31.6% of patients, AST was increased in 35.4% of patients, and bilirubin was increased in 5.1% of patients [14]. Why do COVID-19 patients suffer from digestive system damage? Is the injury caused by SARS-CoV-2 virus directly or by the systemic inflammatory response (SIRS)? We rarely know the mechanism of the digestive system damage in COVID-19 patients. But the knowledge about it is significant for clinical treatment guidance.

In this study, immunohistochemistry was applied to detect the expression of ACE2 protein in the human liver, esophagus, stomach, and colon. The role of ACE2 in the COVID-19 digestive system damage was explored in the study, with the help of relevant references. New strategies for the prevention and treatment of the COVID-19 digestive system organ damage may be provided.

## 2. Materials and Methods

### 2.1. Reagents

Rabbit monoclonal antibody to ACE2 was purchased from the Abcam Company. BSA was bought from the Shanghai Shenggong Biology Co., Ltd. Hematoxylin staining solution was bought from the Beijing Zhongshan Jinqiao Biotechnology Co., Ltd. Powder antigen repair solution (citric acid method), PBS phosphate buffer (powder), ready-to-use immunohistochemical hypersensitive UltraSensitive^TM^ immunohistochemical kit reagent, DAB color kit, and Super PAP Pen Super Immunohistochemical Oil Pen were purchased from the Fuzhou Maixin Biotechnology Co., Ltd.

### 2.2. Specimens

Liver samples were collected from patients with hepatic hemangioma. Esophageal mucosa, gastric mucosa, and colonic mucosa were obtained from tissues biopsied for diagnostic purposes. All the specimens were diagnosed by pathological examination. The mucosal tissues were identified to be liver tissue, esophageal mucosal tissue, gastric tissue, and colonic mucosal tissue, with normal structure by the Department of Pathology of the Affiliated Nanhua Hospital of USC. All the patients had not received any kind of treatment, such as radiotherapy, chemotherapy, and targeted therapy and had not been exposed to any biochemical toxicants. Research followed the tenets of the Declaration of Helsinki. Study protocols were approved by the Institutional Review Board at the Affiliated Nanhua Hospital of University of South China, and study participants underwent informed consent by the treating digestive physician.

### 2.3. Immunohistochemistry

All specimens were fixed by 10% paraformaldehyde solution for about 12–24 hours and embedded by paraffin. Paraffin-embedded tissue sections of 5 *μ*m thick were placed in a 60°C thermostat for 1 hour and hydrated through a series steps of xylene and ethanol baths to water. Deparaffinized sections were boiled in antigen retrieval solution (citric acid method) for 5 min and cooled down for 20 min, and a total of 4 repairs were practiced. In slides were added one drop of peroxidase blocking solution and then washed with hot tap water for 1 min and PBS twice for 3 min each time. After cleaning PBS, slides were incubated with anti-ACE2 antibody and left overnight in 4°C in the refrigerator. After 3 washes with PBS, the sections were incubated with the secondary biotinylated goat anti-rabbit IgG for 20 min at room temperature and rinsed with PBS solution 3 times, 3 minutes each time. Slides were covered totally by the preprepared DAB chromogenic solution and placed in room temperature for color development. When light yellow is observed, slides were rinsed with tap water to stop the chromogenic reaction. The sections were also counterstained with hematoxylin counterstain in the nucleus and mounted with the mounting medium.

### 2.4. Result Judgment of Immunohistochemistry

The expression level of ACE2 was interpreted according to the staining results that were observed by the microscope. If the expression of staining is light yellow, brownish yellow, or tan, then ACE2 is positive. Five observation sections of the high magnification field (×400) were randomly observed to observe the staining. We clarified the staining intensity of the cytoplasm and cell membrane of the stained cells and determined the proportion of stained cells in all tissue cells to level staining. The staining intensity was divided into 0 (no positive cells), 1 (weak staining intensity of light yellow), 2 (moderate staining of brownish yellow), and 3 (strong staining of brownish brown). The percentage of positive staining was scored as 0 (negative), 1 (1–25%), 2 (26–50%), 3 (51–75%), and 4 (76–100%). The staining score was the product of staining intensity and percentage of positive staining. The score of 0 was judged as (−), 1–4 as weakly positive (+), 5–8 as positive (++), and 9–12 as strongly positive (++++). Immunohistochemistry scores were expressed as mean ± standard deviation, the MD ± SD.

## 3. Result

### 3.1. ACE2 Is Expressed in Human Liver Tissues

The positive ACE2 staining in liver tissues is observed brownish yellow. The typical cytoplasmic staining indicates that ACE2 mainly exists in the cytoplasm. No positive staining is found in the cell membrane, while a little staining could be observed in the lumen of vascular endothelial cells and bile ducts. The magnification is 400× (Figures 1(a)–1(c)). According to the immunohistochemical score, three liver tissue specimens were positive (++).

### 3.2. ACE2 Is Expressed in Human Esophageal Mucosal Tissues

ACE2 is observed in the mucosal layer of esophageal tissue with brownish yellow staining. No positive staining was observed in other parts. It is mainly localized in the cytoplasm. The magnification is 400× (Figures 1(d)–1(f)). According to the immunohistochemical score, two cases in the group were positive (++) (Figures 1(d) and 1(e)) and one case was weakly positive (+) (Figure 1(f)).

### 3.3. ACE2 Is Expressed in Human Gastric Mucosal Tissues

If ACE2 is positive in human gastric mucosal tissues, the staining is brownish yellow. All three specimens were obtained from the fundic glands of the gastric mucosal epithelium, and the positive expression is located in the cytoplasm. The magnification is 400× (Figures 1(g)–1(i)). According to the immunohistochemical score, two cases in this group were positive expression (++) (Figures 1(h) and 1(i)) and one showed mild positive (+) (Figure 1(g)).

### 3.4. ACE2 Is Expressed in Human Colonic Mucosal Tissues

ACE2 was observed in colonic tissue with the brownish yellow color. It was located in the cytoplasm. Staining is visible on the brush border of the villi. The magnification is 400× (Figures 1(j)–1(l)). Based on the immunohistochemical score, two of the three specimens in the group showed positive expression (++) (Figures 1(j) and 1(k)) and one showed litter positive (+) (Figure 1(l)).

### 3.5. Grading of Immunohistochemistry

On the basis of Table 1, it can be concluded that the liver tissue got the highest score of ACE2 immunohistochemical staining intensity score, followed by gastric tissue, colonic tissue, and esophageal mucosal tissue.

## 4. Discussion

ACE2 is expressed in many human organs and tissues. Its expression in the lung generally is located in the type II alveolar epithelial cells [15]. Its expression in the kidney is mainly located in renal tubule cells, but the expression cannot be found in the immune cells and epidermal cells of the glomerulus [16]. Some studies have shown that ACE2 is expressed in vascular endothelial cells, arterial smooth muscle cells, and cardiac cells [17]. Significant myocardial injury, including myocardial fibrosis and myocardial hypertrophy, is seen in ACE2 knockout mice [18, 19]. In brain tissue, ACE2 is expressed in a low level with only a small amount of ACE2 expressed in glial cells and neurons of the brain [20].

In addition to the lung, kidney, and heart, ACE2 mRNA is also expressed in digestive organs, mainly in the gallbladder, bile duct, and stomach [21]. Another study shows that the expression level of ACE2 mRNA in the digestive system is higher than that in the lung [22]. The protein expression of ACE2 in the digestive system has not been reported. In this study, the results of immunohistochemistry showed that ACE2 protein was expressed in the liver, stomach, esophagus, and colon. ACE2 expression in the liver was mainly located in the cytoplasm of the liver, and no positive staining was observed on liver cell membrane. Slight staining was observed in the vascular endothelial cells and lumen of the bile ducts. The expression of ACE2 in esophageal mucosa was mainly located in the epithelial cytoplasm, and no positive staining was observed in other sites. ACE2 expression in gastric mucosa was mainly located in the epithelial cytoplasm of gastric fundus gland of gastric mucosa. ACE2 expression in colon tissue was mainly located in the cytoplasm of colon mucosal epithelial cells, and staining was observed in the brush border of villus. The ACE2 immunohistochemical staining strength score was in the order of the liver, stomach, and esophagus, as the weakest staining was observed in the esophageal mucosa. According to the results, ACE2 was expressed in the liver, esophagus, stomach, and colon tissues.

At present, novel coronavirus disease 2019 (COVID-19) that is caused by SARS-CoV-2 still threats human health all over the world. In addition to the lung damage, SARS-CoV-2 also causes damage to organs of other systems, including the digestive system. In the early stage of our study, we found that among the 48 COVID-19 patients in the Hengyang area, 27.1% of the patients developed poor appetite, 8.3% of the patients developed nausea and vomiting, and 14.7% of the patients developed diarrhea. Except for primary liver diseases such as viral hepatitis, ALT was elevated in 22.9% of patients, AST was increased in 20.8% of patients, ALP was increased in 5.4% of patients, and *γ*-GT was increased in 21.6% of patients. It is significant to study the mechanism of the digestive system damage in COVID-19 patients for guiding clinical treatment.

SARS-CoV-2 is a kind of single-stranded RNA virus. Its genome sequence contains 29,891 bases, and its virions are spherical with a diameter of 60–140 nm. There are four kinds of structural proteins in SARS-CoV-2 from the envelope to the virus core, the envelope protein (E protein), spinous process protein (S protein), membrane protein (M protein), and nucleocapsid protein (N protein) [23, 24]. At present, the pathogenesis of COVID-19 mainly includes ACE2-mediated direct damage, cytokine storm, ischemia-hypoxia, and drug damage. Through the autopsy on COVID-19 patients, Wang's team found the apoptosis of the liver cell of COVID-19 patients was significant obvious, and there were typical SARS-CoV-2 virus particles in the liver cells [25]. Another autopsy result showed that there were metamorphosis, necrosis, and exfoliation in some epithelial cells in gastrointestinal mucosa [26]. These findings suggest that the digestive system damage in COVID-19 patients may be caused by viral infection. Therefore, the high expression of ACE2 in the digestive system may suggest that the digestive tract may be the potential route of infection.

The binding of ACE2 and S protein is the first step for the virus to invade cells. The S protein of SARS-CoV-2 envelope is transmembrane glycoprotein that includes two subunits, S1 and S2. The receptor binding domain of S1 subunit mediates the invasion through binding to the host cell receptors, while S2 subunit promotes the fusion of virus and host cell membrane; therefore, it narrows the distance between them [27]. S protein can also be activated by a variety of proteases (such as trypsin and elastase) to promote the formation of syncytium on the cell surface, which is critical for virus invasion. When S protein binds to ACE2 on the cell surface, the former is activated by transmembrane protease serine 2 (TmRSS2), and thus, TMPRSS2S protein and ACE2 constitute protein complex and undergo conformational changes. That divides S protein into S1 and S2 subunits, which are attached to the host cell membrane and undergo membrane fusion, promoting SARS-CoV-2 to invade cells for infection replication [28].

In the COVID-19 treatment studies, targeting ACE2 provides the possibility to prevent the invasion of SARS-CoV-2, while maintaining RAS homeostasis may also help to reduce the damage to the digestive system. In their research, Zhang's team established a colitis mouse model by using dextran sulphate sodium salt to treat ACE2 gene knockout mice and subsequently found that the level of AngII in the damaged colon tissue increased. After using the human recombinant soluble ACE2 (HRSACE2), a lower level of ANGII than before showed up [29]. Therefore, HRSACE2 can maintain the activity of ACE2 of host cell. Previous studies have shown that HRSACE2 combined with SARS-CoV-2 can significantly inhibit virus infection [30]. ACEI and ARB have also been proved; they are effective in alleviating the progression of ARDS [31, 32]. But ACEI and ARB can increase the expression of ACE2, which may promote the invasion of SARS-CoV-2. So that, the use of ACEI and ARB in COVID-19 patients is still controversial. Studies have shown that SARS-CoV-2 monoclonal antibody MAB4A8 can effectively neutralize SARS-CoV-2 and reduce the binding of SARS-CoV-2 and ACE2 [33].

The results of this study showed that ACE2 was expressed in the liver, esophagus, stomach, and colon tissue, which suggests that SARS-CoV-2 may enter the digestive system through ACE2 and cause liver and gastrointestinal damage.

## Figures and Tables

**Figure 1:** (a)–(c) Expression and localization of ACE2 in human liver tissues. (d)–(f) Expression and localization of ACE2 in human esophageal mucosal tissues. (g)–(i) Expression and localization of ACE2 in human gastric mucosal tissues. (j)–(l) Expression and localization of ACE2 in human colonic mucosal tissues. Dewaxed liver tissue sections are treated with rabbit anti-ACE2 antibody for immunohistochemistry. ACE2 expression was analyzed in human liver tissues ((a)–(c)), human esophageal mucosal tissue ((d)–(f)), human gastric mucosal tissues ((g)–(i)), and human colonic mucosal tissues((j)–(l)). Boxed regions in the left of ((a)–(l)) are shown at higher magnification in the right panel (400×).

**Table 1:** Immunohistochemical score of every tissue specimen.

Tissue	Cytoplasm		Average score (MD ± SD)
	Dyeing intensity	Average positive area (%)	
Liver	*M*	86.7	8.00 ± 0.00
Esophageal mucosal	*M*	55.3	5.30 ± 1.15
Gastric mucosal	*M*	56.7	6.00 ± 2.00
Colonic mucosal	*M*	56.7	6.00 ± 3.46

## Data Availability

The data used to support the findings of this study are available from the corresponding author upon request.
